RETRACTED

# Risk Factors for Thyroid Dysfunction in Patients with Advanced Non-Small-Cell Lung Cancer Treated with PD-1 Antibody

**DOI:** 10.1155/2022/9086962

**Published:** 2022-08-12

**Authors:** Junjun Zhang, Jing Lou

**Affiliations:** ^1^Endocrinology Department, Hunan Provincial People's Hospital, The First Affiliated Hospital of Hunan Normal University, Changsha, Hunan 410100, China; ^2^Surgery, Changsha County Maternal and Child Health Care Hospital, Changsha, Hunan 410100, China

## Abstract

**Objective:**

To analyze the health status of thyroid function in patients with advanced non-small-cell lung cancer cured with PD-1 antibody and to explore the risk factors of thyroid dysfunction.

**Methods:**

100 patients from Hunan Provincial People's Hospital with advanced non-small-cell lung cancer hospitalized from January 2021 to March 2022 were selected. All patients were treated with a PD-1 antibody. The differences in sex, age, operation history, chemotherapy history, radiotherapy history, and thyroid nodules between patients with abnormal thyroid function and normal thyroid function after treatment were compared. Moreover, the risk factors of thyroid dysfunction were analyzed.

**Results:**

The proportion of women in the normal thyroid function group was lower compared to the abnormal thyroid function group. And the proportion of patients with the course of the disease within 1 year in the normal thyroid function group was higher compared to the abnormal thyroid function group. The incidence of thyroid color ultrasound nodules in the normal thyroid function group was remarkably higher compared to the abnormal thyroid function group (*P* < 0.05). The proportion of patients with nodules in the abnormal thyroid function group was remarkably higher compared to the normal thyroid function group. Among the 36 patients who developed abnormal thyroid function, the incidence of hyperthyroidism (hyperthyroidism) and subclinical hyperthyroidism (subclinical hyperthyroidism) was 33.33%. The incidence of hypothyroidism (hypothyroidism) and hypothyroidism (subclinical hypothyroidism) was 66.66%. The cumulative incidence rates after 3 cycles, 6 cycles, and 12 cycles were 63.88%, 83.33%, and 94.44%, respectively. T4 and FT3 levels decreased more than the normal group following therapy. The results showed that females, course of disease more than one year, and thyroid nodule were independent risk factors of thyroid dysfunction.

**Conclusion:**

Female gender, disease duration of more than 1 year, and thyroid nodules were independent risk factors for thyroid dysfunction after PD-1 antibody therapy. Therefore, clinical treatment should focus on patients with the above factors, and early intervention should be implemented to avoid the occurrence of thyroid dysfunction after PD-1 antibody treatment.

RETRACTED

## 1. Introduction

In recent years, the incidence and mortality of malignant tumors have increased year by year, which has become a major threat to global human health. According to related research reports, the incidence and mortality of malignant tumors in China are increasing year by year, which has become the leading cause of death of urban residents in China. Chinese patients with lung cancer have one of the highest mortality rates of all malignant tumors. It poses a serious threat to the health and life of patients. Globally, lung cancer kills more than 1.7 million people every year. It is the leading cause of cancer-related deaths. There are about 733,000 new cases and about 591,000 deaths [1–3]. Clinically, lung cancer is divided into small-cell lung cancer and non-small-cell lung cancer. More than 80% of lung cancer is non-small-cell lung carcinoma (NSCLC), which is prone to distant metastasis with a high fatality rate [4]. Early-stage NSCLC patients are typically asymptomatic and most of them are diagnosed late in the process of the disease, missing the ideal time for optimal treatment. In clinic, chemotherapy is often used to treat patients with advanced lung cancer, which can alleviate clinical symptoms and prolong the survival time of patients to some extent [5].

Pemetrexed/docetaxel/gemcitabine/vinorelbine + carboplatin/cisplatin/nedaplatin is a commonly used chemotherapy regimen for lung cancer, but its adverse reactions are large and some patients are poorly tolerated. It can have a negative impact on the prognosis of patients. With the deepening of human understanding of immune regulation technology, tumor therapy has entered a new era [6–8]. The successful targeting and inhibitory effect of immune checkpoint inhibitors make them play a significant role in antitumor therapy. It has been used when treating malignant tumors. It has greatly improved the survival rate of patients and has become the first-line drug when treating malignant tumors. The antitumor effect is that monoclonal autoantibodies against T cell inhibitory receptors include cytotoxic T lymphocyte antigen 4, programmed death 1, and their ligands. These monoclonal antibodies block immune checkpoints and release T cells to fight cancer [9–11]. Immune checkpoints also attach importance to maintaining immune self-tolerance and preventing autoimmune diseases. Immune checkpoint inhibitors can also bring about the activation of autoreactive T cells during antitumor therapy, which leads to unique immune-related adverse events.

At present, seven immunosuppressants have been approved to treat tumors, such as PDL-l (programmed death ligand 1), PD-1 (programmed death receptor 1), CTLA4 (CytotoxicTIymphocyteassociated4) [12, 13]. These nonspecific immune enhancements not only target tumor cell-associated antigens but also attack autoantigens, resulting in immune-related adverse reactions [14, 15]. Immune-related adverse reactions can affect many systems of the body, like the gastrointestinal tract, liver, skin diseases, and endocrine system. If these adverse reactions are not detected and treated in time, the consequences may be fatal. Among them, the highest incidence is endocrine-related immune adverse reactions, which are relatively harmful to the human body because of their irreversibility [16]. Thyroid adverse reactions are the most common in the reports so far. Thyroid dysfunction is mainly related to anti PD-1 therapy and combined anti PD-1 and anti CTLA-4 therapy [17]. Immunosuppressant-related thyroid dysfunction is the most common immune adverse reaction in the endocrine system associated with ICPI, occurring within weeks to months after the initiation of ICPI [18]. It mainly includes hypothyroidism and hyperthyroidism. Hyperthyroidism may be transient, initially manifesting as transient thyrotoxicosis, then transforming into overt or subclinical hypothyroidism, and eventually, thyroid hormone levels return to normal [19]. In severe cases, hypothyroid heart disease may occur; hyperthyroidism may have hypermetabolic symptoms such as fever, profuse sweating, and weight loss. Thyroid storm and thyrotoxic heart disease occur. These symptoms can be life-threatening if not detected in time. The incidence of thyroid dysfunction caused by programmed cell death protein-1 or its ligands is 7–21% and the incidence of cytotoxic T lymphocyte antigen-4 is 0–6%. Among all immunosuppressive monotherapy, programmed death receptor-1 inhibitors are most likely to cause thyroid dysfunction [20]. The research on the mechanism of tumor action of PD-1 inhibitors is becoming more and more thorough and its clinical application will be greatly increased. Understanding the evolution of thyroid diseases can be used to guide patient management, monitoring, and follow up. Based on this, this study aimed to explore the correlation and clinical significance between PD-1 antibody therapy and thyroid dysfunction in patients with advanced non-small-cell lung cancer.

RETRACTED

## 2. Materials and Methods

### 2.1. General Information

One hundred patients from Hunan Provincial People's Hospital with advanced NSCLC hospitalized from January 2021 to March 2022 were cured with a PD-1 antibody. Following treatment, they were assigned into the normal and abnormal groups on whether the thyroid function was normal or not. The baseline data and statistical analysis results are shown in Table 1. We obtained the approval of the Medical Ethics Association at our hospital and all patients provided informed consent.

Selection criteria: (1) NSCLC was diagnosed by pathological biopsy and imaging examination) clinical stage III b ∼ IV with measurable or evaluable tumor lesions; (3) complete medical history and pulmonary imaging data; (4) chemotherapy was the first choice; (5) Karnofsky functional status score ≥60.

Exclusion criteria: (1) patients who were complicated with other malignant tumors; (2) the patients did not follow the indication of chemotherapy; (3) intolerant to therapeutic drugs; (4) Karnofsky functional status score <60; (5) severe history of drug allergy; (6) complicated with autoimmune disease or interstitial pneumonia.

### 2.2. Methods

All selected patients received an intravenous injection of PD-1 inhibitor: (1) 3 mg of papolizumab every 3 weeks; (2) 3 mg/kg of triplizumab every 3 weeks; (3) Sintilimab 200 mg every 3 weeks; (4) Camrelizumab 200 mg every 3 weeks; (5) Tislelizumab 200 mg every 3 weeks. Thyroid function including serum thyroid stimulating hormone (TSH), free thyroxine (FT4), and free triiodothyronine (FT3) was carried out at the end of baseline and 2 treatment cycles. During the trial, the normal or transient changes of TSH and FT4 (shorter than 2 consecutive treatment cycles) were regarded as normal thyroid function groups. 21 days were taken as a trial medication cycle. At least 2 consecutive trial medication cycles with abnormal levels of TSH and FT4 were regarded as thyroid dysfunction group.

### 2.3. Observation Index

#### 2.3.1. Patient Baseline Data Statistics

In the hospital medical record system, the patient's sex, age, course of the disease, medical history, and BMI index were statistically analyzed.

#### 2.3.2. Statistics of Thyroid Function of Patients

After two cycles of treatment, thyroid color Doppler ultrasonography was performed to determine whether there were thyroid nodules. The baseline level of TSH, the incidence of thyroid dysfunction, the onset period, and clinical classification of thyroid function were counted. The thyroid function of the patients was judged according to the levels of serum thyrotropin, free thyroxine, and free triiodothyronine. During the trial, the normal or transient changes of serum thyroid stimulating hormone and free thyroxine (shorter than 2 consecutive treatment cycles) were regarded as normal thyroid function groups.

#### 2.3.3. Correlation Analysis of Factors of Thyroid Dysfunction

The course of the disease, type of solid tumor, medical history, BMI index, thyroid nodules, and TSH baseline level was analyzed by Logistic regression.

RETRACTED

### 2.4. Statistical Analysis

SPSS23.0 statistical software was adopted to process the data. The measurement data were presented as ($\bar{x}$ ± *s*). The group design *t*-test was adopted for the comparison and the analysis of variance was adopted for the comparison between multiple groups. The dun-net-t test was adopted for comparison with the control group. The counting data were presented in the number of cases and the percentage. *χ*^2^ test and multiple Logistic regression were adopted to analyze the risk factors related to the prognosis of children. The difference exhibited statistically significant, and difference was statistically significant (*P* < 0.05).

## 3. Results

### 3.1. Comparison of Baseline Data of Patients

The difference in gender ratio was statistically significant (*P* < 0.05). Among them, the proportion of women in the normal thyroid function group was lower (*P* < 0.05). The proportion of patients with a course of less than 1 year in the normal thyroid function group was remarkably higher compared to the abnormal thyroid function group. All results are shown in Table 1.

### 3.2. Comparison of Thyroid Function

A significant difference was exhibited in the incidence of thyroid nodules (*P* < 0.05). The proportion of nodules in the abnormal thyroid function group was remarkably higher compared to the normal thyroid function group. A total of 36 patients developed thyroid dysfunction. The incidence of hyperthyroidism and hypothyroidism was 33.33%. The incidence of hypothyroidism and hypothyroidism was 66.66%. After 3, 6, and 12 cycles, the cumulative incidence was 63.88%, 83.33%, and 94.44% respectively. No difference was exhibited in the baseline levels of FSH, FT4, and FT3. After treatment, the level of FSH in the abnormal thyroid function group increased remarkably compared with the normal group and the levels of FT4 and FT3 decreased compared with the normal group (*P* < 0.05). All results are shown in Table 2 and Figures 1 and 2.

### 3.3. Correlation Analysis of Factors of Thyroid Dysfunction

Sex, course of the disease, history of operation, history of chemotherapy, history of radiotherapy, BMI index, no thyroid nodule, and baseline TSH level were taken as independent variables (see Table 3). Thyroid dysfunction (no = 0, yes = 1) was taken as the dependent variable to analyze the related factors. The results showed that females, the course of disease more than one year, and thyroid nodules were the independent risk factors of thyroid dysfunction. All results are shown in Table 4.

RETRACTED

## 4. Discussion

According to estimates from my country's Cancer Statistics 2015, there were 4,292,000 new malignant tumor patients in my country in 2015 with an average of about 12,000 newly diagnosed malignant tumor patients every day. The number of cancer deaths was as high as 2,814,000 with an average of more than 7,500 patients per day died of malignant tumors. The vast majority of new cases and deaths from lung cancer occur between 60.74 years old, and it has the highest mortality rate in the population [21–24]. Clinically, tumors are divided into nonsolid tumors and solid tumors [25, 26]. Solid tumors can be detected by clinical CT scanning, B-ultrasound, and X-ray, which can be divided into benign and malignant tumors. The existence of solid tumors has a great impact on patients, seriously reduces the life quality of patients, and threatens their life and health of patients. In the clinical treatment of advanced solid tumors, some antineoplastic drugs are often used to delay the development of patients' conditions and prolong their survival time [27]. Traditional treatment methods such as surgery, chemotherapy, and radiotherapy often cannot significantly improve the survival time of patients with advanced tumors. Therefore, there is an urgent need to find new tumor treatment models. Because of the particularity of the tumor growth environment, it not only depends on its cytokines but also can avoid immune regulation and monitoring through signal pathways. With the development of medical technology in recent years, it has been found that immunotherapy can play a better therapeutic effect when treating the tumor. After surgery, radiotherapy, and chemotherapy, tumor immunotherapy has gradually gained in popularity [28]. After Rosenberg successfully used IL-2 to cure advanced MM patients in 1985, the concept of tumor biological immunotherapy was formally put forward. In recent years, modern biological immunotherapy has become the fourth treatment mode for malignant tumors [29]. Tumor immunotherapy has attracted more and more attention, especially anti PD1/PDL1 antibody, which has achieved great success when treating malignant tumor patients and brought hope to some patients. Programmed death protein belongs to the B7 molecular protein family, which is a type I transmembrane glycoprotein with a molecular weight of 50∼55 kDa [30]. The protein was expressed on DC cells, B cells, T cells, natural killer cells, mononuclear macrophages, tumor cells, and activated vascular endothelial cells. Its ligand PD-L1 is expressed on the surface of malignant melanoma, gastric cancer, esophageal cancer, pancreatic cancer, renal cell carcinoma, breast cancer, lung cancer, and other tumor cells. PD-1 is a kind of immunosuppressive molecule, which can promote the apoptosis of tumor antigen-specific T cells by interacting with PD-L2 and PD-L1. Cancer cells are not monitored by the immune system in the body, so PD-L1 is expressed at significantly higher levels in cancer tissues than in normal tissues. The application of PD-1 antibodies can activate T cells, block PD-L1 and PD-1 pathways, activate the body's immune system, and effectively kill tumor cells [31].

RETRACTED

Thyroid dysfunction is a common immune adverse reaction when treating PD-1. Typical thyrotoxicosis changes from hyperthyroidism to hypothyroidism, or only hypothyroidism. Thyrotoxicosis associated with PD-1 inhibitors is caused by destructive thyroiditis or autoimmunity, destroying thyroid follicular epithelial cells and the release of reserved thyroid hormones, characterized by hyperthyroidism. PD-1 transmembrane receptor in hypothyroidism is an immune checkpoint receptor that can act on activated T cells, B cells, natural killer cells, and macrophages, thus improving the tolerance of the body to autoimmunity [32]. PD-1 can bind to PD-L1 and PD-L2, thus down-regulating the effect of self-antigen on the body and producing tolerance. Cancer cells can overexpress PD-L1 through gene mutation or tumor microenvironment, which can escape the antitumor effect of T cells [33]. Overexpression of PD-L1 can occur in various human cancers. PD-L1 can be expressed not only on tumor cells but also in the process of thyroid inflammation. Recent studies have shown that PD-L1 and PD-L2 have been examined in normal thyroid mRNA and protein levels. This has suggested that the interaction between PD-1-expressing lymphocytes and PDL-expressing thyroid cells allows the thyroid gland to escape autoimmune attacks [34]. The destruction of this interaction caused by PD-1 or PD-L1 antibodies may bring about thyroid autoreactive T and B lymphocyte infiltration, which eventually leads to thyroiditis. Various studies have found that the expression of PD-L1 is increased in chronic lymphocytic thyroiditis and Hashimoto's thyroiditis, indicating that the immune microenvironment provided by chronic inflammation can enhance the expression of PD-L1 [35]. Early studies have found that in CLT60% cytoplasmic PD-L1 positive, 40% cell membrane PD-L1 positive, in HT80% cytoplasmic PD-L1 positive, 20% cell membrane PD-L1 positive, while benign nodules did not detect PD-L1 staining [36]. The presence of CLT and HT affects the expression of PD-L1 in the benign follicular metaplastic epithelium and thyroid papillary carcinoma. At the same time, thyroid staining was performed in 4 patients with diffuse toxic goiter, and no expression of PDL or PD-1 was found. PD-L1 was not detected in the benign thyroid gland and thyroid papillary carcinoma excluding thyroiditis [37]. Significant PD-L1 expression was detected in 2 of 5 CLT patients with PD-L1,5 and HT patients. Thus, the immune microenvironment attaches importance to PD-L1 expression.

RETRACTED

The results showed that females, course of disease more than one year, and thyroid nodule were independent risk factors of thyroid dysfunction. At present, the mechanism of thyroid adverse reactions caused by PD-1 antibody treatment is not clear. Some studies believe that the cause of this adverse reaction may be related to immune-related inflammatory thyroiditis. In the process of treatment, it will not only activate T cells but also affect B cells, thus activating thyroid autoantibodies, leading to inflammatory reactions, resulting in thyroid adverse reactions. Anti PD-1 antibody plays an important role in blocking the PD-1/PD-L1 pathway, which can realize the negative regulation of cellular immunity and reactivate the antitumor effect of T cells. The application of this kind of drug may also enhance the immune-related signal pathway and enhance the immune activity of patients, which can lead to the imbalance of immune tolerance in other normal organs. Then the development of immunotherapy leads to the emergence of inflammatory reaction, which has a great impact on the body of patients [38]. When treating immune checkpoint inhibitors, including the treatment of anti PD-1 antibody and its ligand PD-L1 antibody as well as the treatment of cytotoxic T lymphocyte-associated antigen-4. The adverse reactions are immune-related adverse reactions. The most common adverse conditions in the process of immunotherapy include skin, lung, liver, colon, and endocrine organs. These immune-related adverse reactions bring great pain to patients. There are even some immune adverse reactions that can pose a serious threat to the health and life of patients, including myocarditis and nervous system diseases [39]. It is considered that the occurrence of immune-associated inflammatory thyroiditis may be related to the factors of thyroid adverse reactions during immunotherapy [40]. Thyroid autoantibodies and local histopathology of patients should be studied continuously. In 2017, Mayo Medicine published a study on the mechanism of thyroiditis. Based on this study, it is concluded that autoantibodies have no clear relationship with the mechanism of thyroid destruction but may be related to the pathway mediated by NK cells, T cells, and monocytes [41]. There are changes in thyroid function, although these patients do not need to receive treatment intervention. However, it is still suggested that we should still pay attention to the effect of the drug on endocrine organs when treating PD-1 antibodies and thyroid function should be tested. At present, the mechanism of thyroid adverse reaction caused by PD-1/PD-L1 antibody treatment is not clear. In the process of immunotherapy, hypothyroidism and hyperthyroidism can be caused by abnormal autoimmune regulation [42, 43]. In 2017, the European Congress of Internal Oncology released guidelines on toxicity management related to immunotherapy. According to the guidelines, it is proposed that thyroid diseases mainly include hypothyroidism and hyperthyroidism during anticancer therapy. Hypothyroidism is a more common thyroid disease. In addition, most patients with hyperthyroidism belong to a temporary reaction, and patients with hyperthyroidism may have further hypothyroidism. After the occurrence of hyperthyroidism, the patients should be treated with antithyroid drugs, steroid drugs, or *β*-blockers, especially in patients with obvious symptoms. Patients with subclinical hypothyroidism or hypothyroidism with related fatigue symptoms need to be treated with thyroid hormone replacement therapy for a long time. This study still has some shortcomings. Firstly, the quality of this study is limited due to the small sample size we included in the study. Secondly, this research is a single-center study and our findings are subject to some degree of bias. Therefore, our results may differ from those of large-scale multicenter studies from other academic institutes. This research is still clinically significant and further in-depth investigations will be carried out in the future.

RETRACTED

To sum up, female gender, disease duration of more than 1 year, and thyroid nodules were independent risk factors for thyroid dysfunction after PD-1 antibody therapy. Therefore, clinical treatment should focus on patients with the above factors, and early intervention should be implemented to avoid the occurrence of thyroid dysfunction after PD-1 antibody treatment.

## Figures and Tables

**Figure 1:** Baseline levels of FSH, FT4, and FT3 in two.

**Figure 2:** Levels of FSH, FT4, and FT3 in two groups during treatment.

**Table 1:** Baseline data between two groups of patients (*n*%).

Project		Normal thyroid function group (*n* = 64)	Abnormal thyroid function group (*n* = 36)	*X* ^2^/*t*	*P*
Gender	Male	47	19	4.382	0.036
	Female	17	17		
Age (years)		51.36 ± 3.73	50.86 ± 3.48	0.658	0.511
Course of disease	≥1 year	17	19	6.872	0.008
	<1 year	47	17		
Surgical history		24	12	0.173	0.676
History of chemotherapy		47	29	0.640	0.423
History of radiotherapy		49	32	2.274	0.131
BMI index (kg/m^2^)	<18.5 or >23.9	38	25	1.002	0.316
	18.5∼23.9	26	11		

RETRACTED

**Table 2:** The thyroid function between the two groups.

Project		Normal thyroid function group (*n* = 64)	Abnormal thyroid function group (*n* = 36)	*X* ^2^/*t*	*P*
Thyroid color ultrasonography	No nodules	25	7	4.075	0.044
	Have nodules	39	29		
TSH baseline level		2.12 ± 0.24	2.05 ± 0.31	1.257	0.211
The onset cycle of thyroid dysfunction	Three-week period		23 (63.88%)		
	Six cycles		30 (83.33%)		
	Twelve cycles		34 (94.44%)		
Clinical classification	Hyperthyroidism		8 (22.22%)		
	Hyperthyroidism		4 (11.11%)		
	Hypothyroidism		13 (36.11%)		
	Hypothyroidism		11 (30.55)		

**Table 3:** Assignment of independent variables.

Independent variable	Assignment	Independent variable	Assignment
Gender	Female = 1, Male = 0	History of radiotherapy	Yes = 1, No = 0
Course of disease	Course of disease ≥1 year = 1, Course of disease <1 year = 0	BMI index	<18.5 or >23.9 = 1, 18.5∼23.9 = 0
Surgical history	Yes = 1, No = 0	Thyroid nodules or not	Have nodules = 1, No nodules = 0
History of chemotherapy	Yes = 1, No = 0	Baseline TSH level	Continuous variable

**Table 4:** Correlation analysis of factors of thyroid dysfunction ($\bar{x}$ ± *s*, points).

Project	*β*	Se	*X* ^2^	OR	95% CI	*P*
Female	0.934	0.421	4.922	2.545	1.115–5.808	0.027
Course of disease ≥1 year	1.024	0.471	4.727	2.784	1.106–7.009	0.030
Surgical history	−0.214	0.428	0.250	0.807	0.349–1.868	0.617
History of chemotherapy	0.172	0.372	0.214	1.188	0.573–2.462	0.644
History of radiotherapy	0.119	0.513	0.054	1.126	0.412–3.079	0.817
BMI index	−0.121	0.631	0.037	0.886	0.257–3.052	0.848
Thyroid nodules	2.104	0.621	11.479	8.199	2.427–27.692	0.001
Baseline TSH level	0.324	0.423	0.587	1.383	0.603–3.168	0.444

## Data Availability

The datasets used and analyzed during the current study are available from the corresponding author upon reasonable request.
